# LncRNA *THOR* increases osteosarcoma cell stemness and migration by enhancing SOX9 mRNA stability

**DOI:** 10.1002/2211-5463.12620

**Published:** 2019-03-20

**Authors:** Haojun Wu, Yanxia He, Hang Chen, Yanzhi Liu, Bo Wei, Guanghua Chen, Han Lin, Hao Lin

**Affiliations:** ^1^ The Orthopaedic Center The Affiliated Hospital of Guangdong Medical University Zhanjiang China; ^2^ The Operating Room The Affiliated Hospital of Guangdong Medical University Zhanjiang China; ^3^ Department of Pharmacology The Affiliated Hospital of Guangdong Medical University Zhanjiang China

**Keywords:** cancer stem cell, long non‐coding RNA, osteosarcoma, SOX9, stemness, *THOR*

## Abstract

Although the long non‐coding RNA *THOR* has been reported to promote cancer stem cell expansion in liver cancer and gastric cancer, its effects on osteosarcoma (OS) cells remain unclear. Here, we investigated the roles of *THOR* in the stemness and migration of OS cells. We report that the level of *THOR* is remarkably upregulated in OS cell spheroids compared to that in OS adherent cells. *THOR* overexpression increased spheroid formation ability and aldehyde dehydrogenase 1 (ALDH1) activity in OS adherent cells, and the opposite effect was observed in spheroids with *THOR* knockdown. Additionally, the spheroids formed by OS adherent cells exhibited a stronger migration ability, which was attenuated by *THOR* knockdown, and *THOR* overexpression increased OS cell migration. Mechanistically, mRNA stability, luciferase reporter, and RNA–RNA *in vitro* interaction assays indicated that *THOR* can directly bind to the middle region of the *SOX9* 3′‐untranslated region (UTR), and enhances its mRNA stability, thereby increasing its expression. Notably, *SOX9* knockdown reduced the ability of *THOR* overexpression to promote the stemness of OS cells. These findings indicate that the lncRNA *THOR* can promote the stemness and migration of OS cells by directly binding to the middle region of *SOX9* 3′UTR, thereby enhancing *SOX9* mRNA stability and increasing its expression; thus, we provide information that may be of use in identifying potential targets for OS treatment.

**Abbreviations**
ActD: actinomycin D
ALDH1: aldehyde dehydrogenase 1
CDS: coding sequence
ceRNA: competing endogenous RNA
CSC: cancer stem cell
EMT: epithelial–mesenchymal transition
lncRNA: long non‐coding RNA
MTT: 3‐(4,5‐dimethylthiazol‐2‐yl)‐2,5‐diphenyl‐tetrazolium bromide
OS: osteosarcoma
qRT‐PCR: quantitative real‐time PCR
RIP: RNA immunoprecipitation
UTR: untranslated region

Osteosarcoma (OS) is common in children and adolescents and characterized by a high incidence and early metastasis. Although the 5‐year survival rate of patients treated with chemotherapy and surgery has been increased to 60–70%, there are still some patients with poor efficacy and recurrence, and the metastasis rate is still up to 30–40% 1. Cancer stem cells (CSCs) lead to tumor recurrence and metastasis 2. Thus, it could facilitate OS treatment or prognosis to elucidate the mechanisms contributing to OS cell stemness.

Long non‐coding RNAs (lncRNAs) are a type of RNA with a length of more than 200 nt and without protein‐coding function 3. Compelling evidence indicates that lncRNAs act as important epigenetic regulators during tumor proliferation 4, apoptosis 5, migration 6 and autophagy 7. Additionally, recent work has established the critical roles of lncRNAs in regulating the stemness of cancer cells; for example, the lncRNA *HAND2‐AS1* maintains the cell stemness by interacting with transforming growth factor β1 in non‐small cell lung cancer 8; the lncRNA *ZNF281* level is lower in glioma stem‐like cells and inhibits their self‐renewing and invasion ability 9; and the lncRNA *B4GALT1‐AS1* could recruit HuR to the nucleus and subsequently promote YAP transcriptional activity, which promotes OS cell stemness 10. LncRNA *THOR* was first identified as a conserved cancer RNA with oncogenic roles in 2017 11. A recent study demonstrates that *THOR* promotes cell proliferation and metastasis in hepatocellular carcinoma 12. Notably, *THOR* facilitates liver CSC expansion by activating β‐catenin signaling 13. Importantly, *THOR*‐mediated binding activity could be disrupted by triptonide in human nasopharyngeal carcinoma cell growth 14. Although recent work has shown the promoting effects of *THOR* in OS cells growth 15, *THOR*'s roles in regulating OS cell stemness remain unclear.

A previous study has shown that *THOR* directly targets stemness marker *SOX9*, through which *THOR* promotes the stemness of gastric cancer cells 16, we wonder whether the *THOR*–*SOX9* axis also exists in OS cells and displays similar effects in OS cell stemness and thus promotes OS cell migration. In the present study, we showed that *THOR* facilitated OS cell stemness and migration through directly binding to the transcription factor *SOX9* mRNA.

## Material and methods

### Cells culture

The human OS cell line MG63 was purchased from ATCC (Manassas, VA, USA). MG63 cells were cultured in 1640 medium (Thermo Fisher Scientific, Waltham, MA, USA) containing 2 mm l‐glutamine and 10% FBS (Thermo Fisher Scientific) under a humidified atmosphere with 5% CO_2_ at 37 °C.

### Spheroid formation assay

This process is referred to in a previous study 17. Briefly, OS cells were trypsinized with trypsin–EDTA (Sigma‐Aldrich, St. Louis, MO, USA) and then cultured in Dulbecco's modified Eagle's medium–F12 medium supplemented with B27 (20 ng·mL^−1^) and epidermal growth factor (10 ng·mL^−1^) in non‐adherent 24‐well plates at 500 cells per well for 8 days, after which spheroids > 50 μm were counted. This experiment was performed in triplicate and repeated at least three times independently. For analysis of spheroid activity, spheroids were collected, trypsinized, re‐seeded in plates and followed by lentivirus infection.

### Lentivirus package

*THOR* overexpression and knockdown and *SOX9* knockdown vectors were constructed by GenePharma (Shanghai, China) and designated Lenti‐*THOR*‐knockdown, Lenti‐*THOR* and Lenti‐*SOX9*‐knockdown, respectively. Lentivirus was packaged by GenePharma.

### Quantitative real‐time PCR

Total RNA was extracted from cells using Trizol regent (Thermo Fisher Scientific) following the manufacturer's recommendation. Then cDNA was reversely synthesized using SuperScript™ First‐Strand Synthesis System for RT‐PCR (Thermo Fisher Scientific, Waltham, MA, USA) according to the standard procedure. Quantitative real‐time (qRT)‐PCR was performed on the StepOne Plus PCR system with Hieff™ qPCR SYBR® Green Master Mix (No Rox; YEASEN, Shanghai, China). mRNA expression levels were normalized to glyceraldehyde 3‐phosphate dehydrogenase expression. The relative expression levels of transcripts were calculated using $2^{-\Delta \Delta c_{t}}$ method.

### mRNA stability assay

This experiment was referred to in a previous study 18. Briefly, 5 μg·mL^−1^ of actinomycin D (ActD; Apexbio, Ann Arbor, MI, USA) was added into MG63 cells with or without *THOR* knockdown to block *de novo* RNA synthesis. Cells were harvested, and total RNA was subsequently extracted at the indicated time points and *SOX9* mRNA level was measured by qRT‐PCR. The *SOX9* mRNA half‐life was evaluated relative to the mRNA level before adding ActD.

### RNA–RNA *in vitro* interaction assay

The detailed procedure was referred to in a previous study 16. Briefly, 25 μL of Protein A/G Magnetic Beads (Thermo Fisher Scientific) was washed twice with RNA immunoprecipitation (RIP) wash buffer (Millipore, Billerica, MA, USA) and then incubated with the BrU antibody (ab2284; Abcam, Cambridge, MA, USA) for 1 h at room temperature. After antibody conjugation, beads were washed twice with RIP wash buffer and subsequently resuspended in incubation buffer containing RIP wash buffer, 17.5 mm EDTA (Millipore) and RNase Inhibitor (Millipore). Equal amounts (5 pmol) of BrdU‐labeled RNAs (*THOR*,* THOR*‐Anti‐sense, LacZ) were incubated with beads in incubation buffer for 2 h at 4 °C. Following incubation, 2.5 pmol of the *SOX9* 5′‐untranslated region (UTR), coding sequence (CDS), 3′UTR RNA fragment was individually added into tubes and incubated overnight at 4 °C. After then, beads were digested, RNA was extracted from the supernatant using the miRNeasy kit (Qiagen, Duesseldorf, Germany), and qRT‐PCR was performed to detect *SOX9* 5′UTR, CDS and 3′UTR levels.

### Transwell cell migration assay

Transwell cell migration assay was performed to examine the migration ability of OS adherent cells with *THOR* overexpression or spheroids with *THOR* knockdown. 24‐well MILLIcell Hanging Cell Culture inserts with 8 mm PET (Millipore) were used for a transwell migration assay. The detailed procedure was referred to the previous work 19. Briefly, OS adherent cells or spheroids were trypsinized and re‐seeded in the upper chamber and allowed to migrate for 48 h. The medium containing 20% FBS served as the chemoattractant. Then, the migrated cells were fixed with methyl alcohol for 15 min, stained with 0.1% crystal violet for 30 min at room temperature, and six random fields from each of the triplicate migration assays were counted using a ×40 objective. Finally, cells stained with crystal violet were washed with PBS three times and destained with 30% acetic acid for 10 min to perform a quantification by measuring with a microplate reader (*D*_570nm_) Corning Inc., Corning, NY, USA. The migration index was shown as the ratio of absorbance intensity.

### Western blot

The detailed procedure was mentioned in a previous study 20. Briefly, cells were lysed using lysis buffer (KeyGEN BioTECH, Nanjing, China). Protein concentration was determined using the BCA Protein Assay Kit (KeyGEN BioTECH). 20 μg of protein was separated by 10% SDS/PAGE, then transferred to nitrocellulose membrane (Promega, Madison, WI, USA) and incubated with the primary antibody against *SOX9* (ab185966), which was purchased from Abcam, primary antibodies against Nanog (cat. no. 14295‐1‐AP), aldehyde dehydrogenase 1 (ALDH1) A1 (cat. no. 15910‐1‐AP), E‐cadherin (cat. no. 20874‐1‐AP), vimentin (cat. no. 10366‐1‐AP) and β‐actin (cat. no. 66009‐1‐Ig) were purchased from Proteintech (Wuhan, Hubei, China). The secondary antibodies (cat. no. KGAA35 and cat. no. KGAA37), horseradish peroxidase conjugated, were purchased from KeyGEN BioTECH. Images were developed using New Super ECL (cat. no. KGP1127; KeyGEN BioTECH). Protein expression levels were quantified by density analysis using quantity one (New Brunswick, NJ, USA) Software and normalized to levels of β‐actin.

### Luciferase reporter analysis

*SOX9* 5′UTR, CDS and 3′UTR sequences were cloned into pMIR‐Report vector, designated PMIR‐*SOX9*‐5′UTR, PMIR‐*SOX9*‐CDS and PMIR‐*SOX9*‐3′UTR, respectively. The sequences of different regions on *SOX9* 3′UTR were inserted into pMIR‐Report vector as well, designated as PMIR‐*SOX9*‐3′UTR‐1 (former), PMIR‐*SOX9*‐3′UTR‐2 (middle) and PMIR‐*SOX9*‐3′UTR‐3 (latter). For confirming the *THOR* targeting on *SOX9*, the above mention luciferase reporter vectors were individually co‐transfected as well as Lenti‐*THOR* infection, and β‐gal plasmid into MG63 cells using Lipofectamine 2000 reagent (Thermo Fisher Scientific) following the manufacturer's recommendation. Seventy‐two hours later, cells were lysed using Reporter lysis buffer (cat. no, E397A; Promega Corp.) and luciferase activity was measured using VivoGlo Luciferin kit (cat. no., P1041; Promega Corp.) and normalized to β‐gal activity.

### ALDH1 activity assay

ALDH1 activity was determined in OS adherent cells or spheroids with different treatment using ALDH Activity Assay Kit (Colorimetric; cat. no. KA3742; Abnova, Taipei, Taiwan, China) following the manufacturer's recommendation.

### MTT assay

MG63 adherent cells with or without *THOR* overexpression, and spheroids with or without *THOR* knockdown were seeded into 96‐well plates and treated with cisplatin treatment (50 nm, cat. no. HY‐17394; MedChemExpress, Monmouth Junction, NJ, USA) 21, 22. After 24, 48 and 72 h, 3‐(4,5‐dimethylthiazol‐2‐yl)‐2,5‐diphenyl‐tetrazolium bromide (MTT) was added into the medium with a final concentration of 5 mg·mL^−1^ and cell viability was examined by measuring the absorbance at 570 nm. Each assay was conducted at least three times.

### Statistical analysis

All results were denoted as mean ± SD and analyzed using prism version X (GraphPad Software Inc., La Jolla, CA, USA). Student's *t* test was used to assess the differences between only two groups. Differences between multiple groups were analyzed using one‐way analysis of variance with the Tukey–Kramer *post‐hoc* test. *P* < 0.05 was considered statistically significant.

## Results

### *THOR* positively regulates the stemness of OS cells

Since there are no unique markers for OS CSCs, we collected the spheroids formed by OS adherent cells, which have been confirmed to have a strong stemness 23. Firstly, we detected *THOR* expression in OS adherent cells and spheroids (Fig. 1A). As expected, OS spheroids displayed a higher expression of stemness markers (Fig. 1B) and stronger ALDH1 activity (Fig. 1C). As shown in Fig. 1D, *THOR* expression was remarkably increased in OS cell spheroids relative to OS adherent cells. Then, *THOR* was overexpressed in OS adherent cells and knocked down in OS cell spheroids by lentivirus infection. The infection efficiency was confirmed in OS adherent cells and spheroids, respectively (Fig. 1E). Notably, we found that *THOR* overexpression increased stemness marker (*Nanog* and *ALDH1*) expression (Fig. 1F–H) and *ALDH1* activity (Fig. 1I). Moreover, the capacity of spheroid formation was enhanced by *THOR* overexpression in OS adherent cells, evidenced by the increase of spheroid size (Fig. 1J) and number (Fig. 1K), while *THOR* knockdown exerted opposite effects in OS cell spheroids (Fig. 1G–K). Thus, these results indicate that *THOR* is positively correlated with the stemness of OS cells.

**Figure 1:** *THOR* positively regulates the stemness of OS cells. (A) Representative picture of spheroids formed by MG63 cells. (B) mRNA levels of stemness markers (*Nanog* and *ALDH1*) were examined in MG63 adherent cells and spheroids. (C) *ALDH1* activity was determined in MG63 adherent cells and spheroids. (D) *THOR* level was detected in MG63 adherent cells and spheroids. (E) The infection efficiency of Lenti‐*THOR* and Lenti‐*THOR*‐knockdown was evaluated in MG63 adherent cells and spheroids, respectively. (F) mRNA levels of stemness markers (*Nanog* and *ALDH1*) were examined in MG63 cells with or without *THOR* overexpression. (G) mRNA levels of stemness markers (*Nanog* and *ALDH1*) were measured in MG63 spheroids with or without *THOR* knockdown. (H) Protein levels of stemness markers (Nanog and ALDH1) were determined in cells and spheroids described in (F,G). (I) ALDH1 activity was determined in cells and spheroids depicted in (F,G). (J,K) Spheroid formation ability was evaluated in cells and spheroids described in (F,G) through measuring the spheroids size (J) and number (K). Difference was assessed using one‐way ANOVA with the Tukey–Kramer *post hoc* test. Data are presented as the mean ± SD, *n* ≥ 3, **P < 0.01 *vs* Control. Scale bar, 50 μm.

### *THOR* positively regulates the migration ability and epithelial–mesenchymal transition process of OS cells

Since CSCs contribute to tumor metastasis, we further evaluated *THOR* effects on the migration ability and the epithelial–mesenchymal transition (EMT) process of OS cells. Notably, OS cell spheroids exhibited a stronger migration ability than OS adherent cells (Fig. 2A,B), and the EMT process was promoted in OS cell spheroids, as evidenced by increased *vimentin* expression (a mesenchymal marker) and decreased *E‐cadherin* expression (an epithelial marker; Fig. 2C,D). Additionally, *THOR* overexpression promoted the migration ability of OS adherent cells (Fig. 2E,F) and facilitated the EMT process characterized as increased vimentin expression (a mesenchymal marker) and decreased E‐cadherin expression (an epithelial marker; Fig. 2G–I), while *THOR* knockdown exerted opposite effects in OS cell spheroids (Fig. 2E–I).

**Figure 2:** *THOR* positively regulates the migration ability and EMT process of OS cells. (A,B) The migration ability was detected in MG63 adherent cells and spheroids by transwell migration assay (A) and quantified (B). (C,D) EMT marker (*vimentin* and *E‐cadherin*) expression was examined in MG63 adherent cells and spheroids. (E,F) Migration ability was determined in MG63 adherent cells with or without *THOR* overexpression, and spheroids with or without *THOR* knockdown by transwell migration assay (E) and quantified (F). (G) mRNA levels of EMT markers (*vimentin* and *E‐cadherin*) were determined in MG63 cells with or without *THOR* overexpression. (H) mRNA levels of EMT markers (*vimentin* and *E‐cadherin*) were examined in MG63 spheroids with or without *THOR* knockdown. (I) Protein levels of EMT markers were measured in cells and spheroids depicted in (G,H). The difference was assayed using one‐way ANOVA with the Tukey–Kramer *post hoc* test. Data are presented as the mean ± SD, *n* ≥ 3, **P < 0.01 *vs* Control. Scale bar, 200 μm.

### *THOR* enhances *SOX9* mRNA stability by directly binding to the middle region of *SOX9* mRNA 3′UTR

We further determined the mechanisms underlying *THOR*‐mediated promotional effects on OS cell stemness. As a previous study has shown direct binding of *THOR* to *SOX9* mRNA, which is responsible for gastric cancer cell stemness 24, we assume that this *THOR*–*SOX9* regulatory axis exists in OS cells as well. Firstly, when *THOR* was overexpressed in OS cells and then ActD was added into the medium to block mRNA *de novo* synthesis, we found that the *SOX9* mRNA decay rate was slower in OS cells with *THOR* overexpression (Fig. 3A). Notably, the *SOX9* mRNA level was upregulated in OS cell spheroids (Fig. 3B) and *SOX9* mRNA decay rate was faster in OS cell spheroids with *THOR* knockdown (Fig. 3C). Further, a luciferase reporter assay demonstrated that *THOR* overexpression enhanced PMIR‐*SOX9*‐3′UTR activity, but had no effects on the activities of PMIR‐*SOX9*‐CDS and PMIR‐*SOX9*‐5′UTR (Fig. 3D). Additionally, an RNA–RNA *in vitro* assay further clarified the direct binding of *THOR* to *SOX9* 3′UTR in OS cells (Fig. 3E). Moreover, we divided the *SOX9* 3′UTR into three parts designated PMIR‐*SOX9*‐3′UTR‐1, PMIR‐*SOX9*‐3′UTR‐2 and PMIR‐*SOX9*‐3′UTR‐3 (Fig. 3F). A luciferase reporter assay indicated that *THOR* overexpression enhanced PMIR‐*SOX9*‐3′UTR‐2 activity, while PMIR‐*SOX9*‐3′UTR‐1 and PMIR‐*SOX9*‐3′UTR‐3 activities were unaffected (Fig. 3G). What is more, *SOX9* expression was increased in OS adherent cells with *THOR* overexpression and decreased in OS cell spheroids with *THOR* knockdown (Fig. 3H,I). These findings suggest the direct binding of *THOR* to the middle region of *SOX9*, which increases *SOX9* expression.

**Figure 3:** *THOR* enhances *SOX9* mRNA stability by directly binding to the middle region of *SOX9* mRNA 3′UTR. (A) *SOX9* mRNA stability was tested in MG63 cells with or without *THOR* overexpression. (B) *SOX9* mRNA level was measured in MG63 adherent cells and spheroids. (C) *SOX9* mRNA stability was measured in MG63 spheroids with or without *THOR* knockdown. (D) Luciferase activity of vector containing different regions of *SOX9* was measured in cells with or without *THOR* overexpression. (E) The *THOR*–*SOX9*‐3′UTR interaction was confirmed using an *in vitro* RNA–RNA interaction assay. (F) *SOX9* 3′UTR was divided into three parts as shown in diagram. (G) The luciferase activity of vectors containing different regions of *SOX9* 3′UTR was determined in MG63 cells with or without *THOR* overexpression. (H,I) *SOX9* expression was examined in MG63 adherent cells with or without *THOR* overexpression, and MG63 spheroids with or without *THOR* knockdown. The difference was assayed using one‐way ANOVA with the Tukey–Kramer *post hoc* test. Data are presented as the mean ± SD, *n* ≥ 3, **P < 0.01 *vs* Control.

### *THOR* promotes the stemness of OS cells through *SOX9*

Then, we determined whether *THOR*‐mediated promoting effects on OS cell stemness are dependent on *SOX9*. *SOX9* was knocked down in MG63 cells with *THOR* overexpression, and stemness marker expression was subsequently examined. As shown in Fig. 4A,B, *SOX9* knockdown attenuated or even reversed the *THOR* overexpression‐induced promoting effects on stemness marker expression. Additionally, the enhanced *ALDH1* activity and spheroid formation mediated by *THOR* overexpression were partially abrogated by *SOX9* knockdown (Fig. 4C–E). qRT‐PCR and western blot analysis were performed to evaluate *SOX9* knockdown efficiency (Fig. 4F,G). Additionally, the promoting effects on OS cell migration mediated by *THOR* overexpression were reduced by *SOX9* knockdown as well (Fig. 4H,I).

**Figure 4:** *THOR* promotes the stemness of OS cells through *SOX9*. (A,B) Stemness marker (*Nanog* and *ALDH1*) expression was detected in MG63 cells with *THOR* overexpression plus *SOX9* knockdown or not. (C) ALDH1 activity was measured in cells described in (A). (D,E) Spheroid formation capacity was evaluated in cells depicted in (A). (F,G) *SOX9* expression was examined in cells described in (A). (H,I) The migration ability was determined in cells depicted in (A) and quantified (I). The difference was assayed using one‐way ANOVA with the Tukey–Kramer *post hoc* test. Data are presented as the mean ± SD, *n* ≥ 3, *P < 0.05, **P < 0.01 *vs* Control. Scale bar, 50 μm (D).

### The *THOR*–*SOX9* axis reduces cisplatin sensitivity in OS cells

Finally, since CSCs could lead to chemoresistance, we investigated the effects of the *THOR*–*SOX9* axis on cisplatin resistance in MG63 cells. MG63 cells with or without *THOR* overexpression were treated with cisplatin (50 nm), and cell viability was subsequently determined. As expected, *THOR* overexpression significantly decreased cisplatin sensitivity of MG63 cells, and this effect was partially abrogated by *SOX9* knockdown (Fig. 5A). Additionally, MG63 cell spheroids exhibited a remarkable decrease of cisplatin sensitivity relative to MG63 adherent cells (Fig. 5B). Importantly, *THOR* knockdown facilitated cisplatin sensitivity of MG63 cell spheroids (Fig. 5C). Notably, ectopic expression of *THOR* alone had no effects on the viability of MG63 adherent cells and spheroids. As a result, these results suggest that the *THOR*–*SOX9* axis could confer cisplatin resistance in OS cells.

**Figure 5:** *THOR*–*SOX9* axis reduces cisplatin sensitivity in OS cells. (A) M63 cells with or without *THOR* overexpression were treated with cisplatin, and their viability was measured by MTT assay. (B) M63 adherent cells and spheroids were treated with cisplatin followed by determining their viability. (C) MG63 spheroids with or without *THOR* knockdown were treated with cisplatin and their viability was determined by MTT assay. The difference was assessed using one‐way ANOVA with the Tukey–Kramer *post hoc* test. Data are presented as the mean ± SD, *n* ≥ 3, **P < 0.01 *vs* Control.

## Discussion

Treatment for OS patients involves multiple chemotherapies, which have remained the main treatment method over the past decades although they are largely ineffective and there are toxic effects 25. As CSCs are the critical promoter of tumor progression, the genetic and epigenetic alterations and the underlying mechanisms of CSC expansion should be intensively explored. Here, we found that the lncRNA *THOR* was remarkably increased in OS cell spheroids, which are enriched in CSCs. Further experiments demonstrated that *THOR* positively regulated stemness marker expression, *ALDH1* activity and spheroid formation in OS adherent cells and spheroids. Our study facilitates the understanding of *THOR* upregulation in OS cell progression.

Over the past several years, lncRNAs have been confirmed as fulfilling their functions through acting as competing endogenous RNAs (ceRNAs) to inhibit miRNA activity; for example the lncRNA *MALAT1* induces breast cancer cell migration and invasion by acting as a ceRNA for *cdc42* 26. Pseudogene *CYP4Z2P* acts as a ceRNA for its parental gene *CYP4Z1* to promote breast cancer angiogenesis 20. Recent studies have shown that many lncRNAs exert their functions through specifically interacting with other cellular factors, such as protein 27, DNA 28 and mRNA 16. Here, RNA–RNA *in vitro* interaction and luciferase reporter analysis confirmed the direct binding of *THOR* to *SOX9* 3′UTR; this is consistent with previous work 16. Although the *THOR*–*SOX9* interaction has been revealed previously 24, we specified the direct binding of *THOR* to the middle region of *SOX9* 3′UTR in this work. Notably, we found that the middle region of *SOX9* 3′UTR holds more potential binding sites for miRNAs than the other two regions (data not shown), and this suggests that *THOR* might promote *SOX9* mRNA stability and its expression by competitively binding to *SOX9* 3′UTR with miRNAs. However, this speculation and the detailed binding sites are still undetermined.

Notably, we found that *THOR* fulfills its function in a *SOX9*‐dependent manner. However, we cannot exclude that other factors are involved in *THOR*‐mediated effects, and elucidating the molecular mechanisms underlying the oncogenic roles of *THOR* requires further effort. As far as we know, this work is the first to reveal *THOR*'s roles in OS cell progression. Moreover, it would facilitate the study of *THOR*'s critical roles in OS progression to explore the upstream effectors of *THOR*.

In conclusion, we have revealed the key functions of *THOR* in OS cell stemness and migration *in vitro*. Notably, we have provided evidence showing the direct binding of *THOR* to the middle region of *SOX9* 3′UTR. Although *in vivo* experiments should be carried out to confirm this *THOR*–*SOX9* axis in OS, our results suggest that *THOR* and *SOX9* in combination may be valuable prognostic predictors for OS and the *THOR*–*SOX9* axis appears to be a promising target for OS therapy.

## Authors contributions

HW and YH conceived and designed the project; HW, YH, HC and YL acquired the data; YL, BW, GC and HL analyzed and interpreted the data; and HW, YH and HC wrote the paper.

## Conflicts of interest

The authors declare no conflict of interest.
